The article "Internet-Facilitated, Voluntary Counseling and Testing (VCT) Clinic-Based HIV Testing among Men Who Have Sex with Men in China" was published in 2013. Journal: PLoS One.

# Internet-Facilitated, Voluntary Counseling and Testing (VCT) Clinic-Based HIV Testing among Men Who Have Sex with Men in China

**DOI:** 10.1371/journal.pone.0051919

**Published:** 2013-02-13

**Authors:** Huachun Zou, Zunyou Wu, Jianping Yu, Min Li, Muhtar Ablimit, Fan Li, Katharine Poundstone

**Affiliations:** 1 Division of Health Education and Behavioral Intervention, National Center for AIDS/STD Control and Prevention, Chinese Center for Disease Control and Prevention, Beijing, China; 2 Sexual Health Unit, School of Population Health, University of Melbourne, Victoria, Australia; 3 Division of AIDS/STD, Xicheng District Center for Disease Control and Prevention, Beijing, China; 4 Center for AIDS/STD Control and Prevention, Xingjiang Uyghur Autonomous Region Center for Disease Control and Prevention, Urumqi, China; University of Washington, United States of America

## Abstract

**Objective:**

To explore the feasibility of using Internet outreach to encourage men who have sex with men (MSM) to get tested for HIV at voluntary counseling and testing (VCT) clinics in Beijing and Urumqi, China.

**Methods:**

From June to August 2007, two volunteers contacted MSM using instant messaging, online chat rooms, mobile phone, and e-mail (active recruitment). Banners with study information were put at the front pages of three major Chinese gay websites (passive recruitment). Those contacted were offered a modest financial incentive to seek HIV testing at existing VCT clinics. Those who subsequently sought HIV testing services at VCT clinics and provided informed consent completed a questionnaire and a blood draw to test for HIV and syphilis.

**Results:**

A total of 3,332 MSM were contacted and 429 attended VCT clinics. One out of every 4 men that were recruited through instant messaging actually went for HIV testing, while the recruitment yields for online gay chat rooms, mobile phone contact, and email were 1∶6, 1∶10, and 1∶140, respectively. The majority of participants (80%, 317/399) reported being motivated to seek HIV testing out of concern for their health, and only 3% (11/399) reported being motivated by the financial incentive. Active recruitment tend to recruit MSM who are younger (X^2^ = 11.400, *P* = 0.001), never tested for HIV (X^2^ = 4.281, *P* = 0.039), tested less often (X^2^ = 5.638, *P* = 0.018).

**Conclusion:**

Internet outreach is a promising way to encourage MSM to seek HIV testing at existing VCT clinics. Active recruitment can target MSM who are younger, never tested for HIV and tested less often.

## Introduction

The number of men who have sex with men (MSM) in China is large. Recent census data indicates that there are 480 million males between the ages of 15 and 59 in China [1]. Previous surveys have suggested that between 2–5% of sexually active Chinese males have had sex with another man at least once in their lives [2], [3], which suggests that the population size of MSM in China may be between 9.6 and 24 million people [4].

HIV prevalence among men who have sex with men (MSM) in China is rising at an alarming rate. In Beijing, HIV prevalence rose from 0.4% in 2004 to 5.8% in 2006 [5]. In Chongqing, it rose from 8.5% [6] in 2007 to 16.8% [7] in 2009. In large cities such as Chongqing, Kunming and Chengdu, HIV prevalence among MSM is now over 9% [6], [8], [9]. Nationwide, the estimated HIV prevalence among MSM was 5% in 2009, far exceeding the general population prevalence rate of 0.05% [10].

The increase in HIV among MSM in China is a reflection of a sexual revolution that has been taking place in China over the past decade [11]. With economic development, urbanization and increased social openness about sexuality, MSM communities have started to grow all across China, and particularly in urban areas. There are no laws against homosexuality in China, and MSM is socially accepted to a greater degree than in other parts of the world. Despite greater social openness about sexuality compared with the past, however, HIV stigma is a major barrier to HIV testing in China, including among MSM [12].

Awareness of HIV status has been shown to help increase condom use and other safer sexual behaviors [13], [14]. However, despite the fact that HIV testing services are widely available, HIV testing rates among MSM in China remain low [4]. China's 2010 United Nations General Assembly Special Session (UNGASS) report indicated that less than half of MSM in China had been tested for HIV in the past 12 months and knew their HIV test result [10]. More effective ways to reach MSM and encourage them to seek HIV testing are urgently needed as part of a comprehensive response to HIV among MSM. The Chinese government recognizes this, and in its ‘Plan for HIV/AIDS Prevention and Control among Men Who Have Sex with Men in China, 2007–2010’, it called on the public health community to use the Internet, telephone hotlines and VCT clinics to scale up HIV testing services for MSM [15].

Internet outreach is a promising way to reach MSM, since many MSM actively use the Internet for social and sexual networking [16]–[18]. The Internet has also been shown to be a good platform to target MSM and carry out HIV and sexually transmitted infection (STI) prevention programs. For example, the Internet was used in San Francisco for partner notification of STIs among MSM [19]; online video-based intervention was adopted to increase HIV testing in MSM in Peru [20]; a web-based cognitive behavioral skills training and motivational enhancement was shown to be effective in reducing sexual risk in MSM in Seattle [21]; and a culturally congruent intervention was shown to be effective in promoting HIV testing among MSM within existing Internet chat rooms [22]. The Internet also offers ways to target otherwise difficult-to-reach sub-populations, such as MSM living in rural and remote areas [17], [23], [24]. The applicability of these prior approaches to the Chinese context remains to be determined, and this is why we set out to determine the feasibility of internet outreach to MSM in the Chinese setting.

The number of gay websites in China is large and still growing. Using the Internet to publicize HIV testing services may encourage more MSM to get tested for HIV and become aware of their HIV status. Therefore, we set out to assess the feasibility of Internet outreach in encouraging MSM to seek existing HIV testing services at VCT clinics in two urban settings: Beijing and Urumqi, China.

## Methods

### Internet outreach

From June to August 2007, two trained MSM community volunteers used the Internet to reach out to MSM and encourage them to seek HIV testing at VCT clinics. One volunteer was based in Urumqi, and the other volunteer was based in Beijing. Each spent 4 hours doing Internet outreach every day, from 6 pm to 10 pm local time, over a period of 30 days.

### Passive Internet outreach

In consultation with MSM community members, a banner was placed on the front pages of a national gay website and three Chinese MSM volunteer websites (http://www.aibai.com; http://www.gengle.net; http://www.hivolunt.com) two weeks prior to the commencement of the study. The banner was an advertisement for the study that read “Health check-up for gay men in Beijing and Urumqi.” Upon clicking the banner, users were directed to a web page with information about the study, including: the incentive offered for HIV testing (CNY 50, ∼USD $7 at the time of study); the addresses and phone numbers for the two participating local VCT clinics; directions to local VCT clinics; how to contact the research team; and the duration of the study. The two volunteers took phone calls from MSM who learned about the study and made appointments for individuals interested in participating.

### Active Internet outreach

The two volunteers abstracted contact information for MSM in Beijing and Urumqi who had posted to three major national gay partner-seeking websites (http://www.pybk.net; http://www.gengle.net; http://www.boysky.com). Information abstracted from these three websites included nicknames, age, current residence, permanent residence, and contact information, including mobile phone numbers, QQ number (instant messaging software, Tencent, China), and email address. The volunteers then used a standardized script to reach out via mobile phone, QQ and e-mail:

Hello. We are volunteers with the Chinese Center for Disease Control and Prevention (CDC). We are doing a health check for gay men at *** (a local CDC VCT clinic). We got your contact number from *** (a gay website). We would like to invite you to participate in this health check, and we provide free testing for HIV and syphilis. We will offer free condoms, lubricant and 50 Chinese Yuan (∼US $7) as a reimbursement for your time.

The volunteers answered questions and booked appointments for those who wished to receive the health check.

The trained community MSM volunteers also chatted with MSM via a Xinjiang-based gay online chatroom (http://www.xj169.com, now defunct). In the chatroom, users can choose to talk to all those logged in, or to specific individuals. Every 5 minutes, the volunteers manually posted the same sentence that all men in the chat room could see:

Hi. We are from the Chinese CDC. We are doing a health-check for gay men in *** (a local CDC VCT clinic). You can get free HIV test, condoms and lubricant and 50 Chinese RMB worth of reimbursement. Please add our QQ *** or call us at *** or send us an email at*** if you are interested!

If someone showed interest by initiating a chat, the volunteer would answer their questions in the chat room. Individuals could also make contact later via QQ or email.

### Study Eligibility

Eligible participants included men aged 18 or older who had had sex with another man or who expressed the desire to have sex with another man.

### Interview, testing and counseling

All MSM who expressed an interest in participating in the study were invited to attend a local VCT clinic in either Beijing or Urumqi for HIV testing. In Beijing, referrals were made to the Xicheng District Center for Disease Control and Prevention (CDC). In Urumqi, referrals were made to the Xinjiang Uighur Autonomous Region CDC.

Those who came in for HIV testing were told about the study and asked to provide informed consent for participation. Pre-test counseling was provided before HIV testing, and post-test counseling was provided when participants received their test results. A nurse collected an intravenous blood sample from each participant for HIV and syphilis antibody testing. Participants were then interviewed face-to-face by trained interviewers. Subjects were surveyed about their socio-demographic characteristics, Internet use, HIV-related sexual behaviors, routes of recruitment and satisfaction with Internet outreach. The results of serological lab testing for HIV and syphilis have been reported previously, along with procedures for post-test counseling and referrals [25].

All participants were provided 50 Chinese RMB (∼US $7) as compensation for their time and local transportation costs. In addition, participants were provided with free condoms, lubricant and MSM health brochures.

### Ethics Review

Trained investigators explained to participants the aim, process, benefits and potential risks of participation of the study before obtaining informed consent. Participants were informed that survey participation was anonymous and voluntary, and that they had the right to discontinue participation at any time. Approval for the study was obtained from the Institutional Review Board (IRB) of the National Center for AIDS/STD Control and Prevention, China CDC, Beijing, China.

### Data Analysis

To determine which recruitment route was most effective at encouraging MSM to receive HIV testing, we calculated the percentage of participants who completed HIV testing by the route of recruitment (QQ, online gay chat room, mobile phone, and e-mail) and compared the proportions using the Chi-square test. To assess the effectiveness of passive versus active recruiting, for each route of recruitment, we also calculated the ratio of those contacted to those who actually completed the study visit, and we compared these proportions using the Chi-square test. EpiData 3.0 was used for double data entry and for validation of the data. Data analysis was performed using SPSS 19.0.

## Results

A total of 3,332 MSM were contacted by two volunteers over the two-month study period, and 429 MSM were recruited into the study. Among the 429 MSM recruited, 420 received HIV and syphilis testing (97.9%), and 399 completed the study questionnaire (93.0%). Most participants were young, well educated, never married, and identified as homosexual (Table 1). In Beijing, a greater proportion of participants reported not being a local resident compared with participants in Urumqi (75.6% versus 49.7%, p<0.001). In addition, participants in Beijing reported higher incomes compared with participants in Urumqi, as consistent with the higher cost of living and level of economic development in Beijing versus Urumqi. Participants from the two cities also differed significantly in self-reported occupation, with more participants in Beijing reporting work as an office clerk (106/254, 41.7%) compared with those in Urumqi (43/145, 29.3%).

**Table 1:** Characteristics of Study Participants.

Characteristics	N (%)^a^	Beijing (%)^a^	Urumqi (%)^a^	*P* d
Age, years (median age = 25 years)				0.900
18–24	171 (42.9)	109 (42.9)	62 (42.8)	
25–29	123 (30.8)	76 (29.9)	47 (32.4)	
30–39	88 (22.1)	57 (22.4)	31 (21.4)	
40–56	17 (4.3)	12 (4.7)	5 (3.4)	
Marital status				0.307
Never married	334 (83.7)	209 (82.3)	125 (86.2)	
Ever married	65 (16.3)	45 (11.3)	20 (13.8)	
Education				0.084
Junior high school or less	16 (4.0)	14 (5.5)	2 (1.4)	
Senior high school	93 (23.3)	62 (24.4)	31 (21.4)	
College or more	290	178	112	
Beijing/Urumqi local resident				<0.001
Yes	135 (33.8)	62 (24.4)	73 (50.3)	
No	264 (66.2)	192 (75.6)	72 (49.7)	
Ethnicity				0.577
Han	362 (90.7)	232 (91.3)	130 (89.7)	
Other^b^	37 (9.3)	22 (8.7)	15 (10.3)	
Salary (RMB)^c^				<0.001
<500	84 (21.1)	44 (17.3)	40 (27.6)	
500-	40 (10.0)	16 (6.3)	24 (16.6)	
1000-	119 (29.8)	68 (26.8)	51 (35.2)	
2000-	156 (39.1)	126 (49.6)	30 (20.7)	
Self reported sexual orientation				0.596^e^
Homosexual	283 (70.9)	180 (70.9)	103 (71.0)	
Heterosexual	74 (18.5)	50 (19.7)	24 (16.6)	
Bisexual	1 (0.3)	1 (0.4)	0 (0.0)	
Undecided	41 (10.3)	23 (9.1)	18 (12.4)	
Occupation				0.014
Office clerk	149 (37.3)	106 (41.7)	43 (29.3)	
Student	93 (23.3)	53 (20.9)	40 (27.6)	
Civil servant	20 (5.0)	7 (2.8)	13 (9.0)	
Other	120 (30.1)	77 (30.3)	43 (29.7)	
Unemployed	17 (4.3)	11 (4.3)	6 (4.1)	

Note:

a Proportions were analyzed based on data of the 399 men who completed a questionnaire;

b Other ethnicities included Uighur, Kazak, Hui and Manchu;

c The currency exchange rate was 7 RMB equaled approximately 1 USD at the time of the study;

d P value from Chi-square test;

e P value from Fisher's exact test.

### Route of recruitment

Among study participants, 35.7% (153/399) were recruited through banners posted on gay websites, 18.6% (80/399) were recruited from gay chat rooms and 41.6% (166/399) were recruited by other routes, including QQ, mobile phone, email and word-of-mouth. Over one quarter (27.4%, 46/168) of men that were approached through QQ actually participated in the study. One in six men contacted via online gay chat room actually attended for the study, the figure for using mobile phone and email were 1∶10 and 1∶140, respectively (Table 2). In Beijing, the majority of participants recruited were recruited through banners on gay websites (49.2% of recruitment), while in Urumqi, the majority of participants were recruited through online gay chat rooms (55.2% of recruitment).

**Table 2:** Routes of recruitment of MSM.

	Total				Beijing				Urumqi			
Route of recruitment	No. Contacted	No. Tested	Proportion of recruitment (%)^a^	Ratio Contacted: Tested	No. Contacted	No. Tested	Proportion of recruitment (%)^a^	Ratio Contacted: Tested	No. Contacted	No. Tested	Proportion of recruitment (%)^a^	Ratio Contacted: Tested
Banner on MSM website	n/a	153	38.3	n/a	n/a	125	49.2	n/a	n/a	28	19.3	n/a
QQ	168	46	11.5	4:1	111	38	15.0	3:1	57	8	5.5	7:1
Online gay chat rooms	458	80	20.1	6:1	n/a	n/a	n/a	n/a	458	80	55.2	6:1
Mobile phone	328	33	8.3	10:1	185	25	9.8	7:1	143	8	5.5	18:1
Email	2378	17	4.3	140:1	1671	15	5.9	111:1	707	2	1.4	354:1
Word of mouth	n/a	70	17.5	n/a	n/a	51	20.1	n/a	n/a	19	13.1	n/a
TOTAL		399	100%			254	100%			145	100%	

Note: “n/a” indicates “not available”.

a : proportion of 399 MSM who provided blood sample and finished a questionnaire.

### HIV testing experiences

Among the 399 participants who provided a blood sample and completed the study questionnaire, 52.1% (208/399) had never been tested for HIV prior to the study. Among those who had been tested for HIV previously, the median time from last HIV test was 9 months, and over one third (67/191) had not been tested in the past 12 months. For MSM who had a sexual history of 5 years or more, during the past 5 years, 55.8% (110/197) had been tested for HIV, and the median number of tests received was 2. A small fraction (7.3%, 8/110) had been tested for HIV 5 times or more.

Among the 420 participants who provided a blood sample, 4.8% (20/420) tested HIV-positive. Among the 19 participants who tested HIV-positive and completed the study questionnaire, 42.1% (8/19) had ever tested for HIV before the study, and 87.5% (7/8) had seroconverted since the time of their last HIV test. Among the HIV-positive MSM who had never been tested for HIV or who had a negative result at their last HIV test, 44.4% (8/18) perceived that they were at very low or no risk of HIV infection.

Among participants who had previously been tested for HIV, over two thirds (67.5%, 129/191) had had their most recent HIV test in a hospital where they had to pay for the test; 22.5% (43/191) had received HIV testing in a VCT clinic; and 9.9% (19/191) had tested in other venues. Nearly all (99.0%, 395/399) reported that they would be more willing to test for HIV if condoms and lubricant are provided. Over two thirds (67.9%, 271/399) reported that they prefer walk-in HIV testing to appointment-based testing (Table 3 and Table 4).

**Table 3:** HIV testing history, perception of risk and HIV result among MSM.

Variable	Total		Beijing		Urumqi		*P* a
	n	%	n	%	n	%	
Ever tested for HIV							0.001
Yes	191	47.9	137	53.9	54	37.2	
No	208	52.1	117	46.1	91	62.8	
Self perception of HIV risk							0.976
Very low or none	70	17.5	46	18.1	24	16.6	
Low	167	41.9	104	40.9	63	43.4	
High	65	16.3	43	16.9	22	15.2	
Very high	13	3.3	8	3.1	5	3.4	
Not sure	84	21.1	53	20.9	31	21.4	
Will you be more willing to test for HIV if condom/lube provided?							1.000^b^
Yes	395	99.0	251	98.8	144	99.3	
No	4	1.0	3	1.2	1	0.7	
Do you prefer appointment or walk-in HIV testing?							0.003
Appointment	128	32.0	95	37.4	33	22.8	
Walk-in	271	68.0	159	62.6	112	77.2	
HIV result from this study							0.732
Positive	20	4.8	12	4.8	8	5.6	
Negative	400	95.2	236	95.2	134	94.4	

**Note:**

a P value from Chi-square test.

b P value from Fisher's exact test.

**Table 4:** HIV testing experience among MSM who have tested for HIV before study.

Variable	Total		Beijing		Urumqi		*P* a
	n	%	n	%	n	%	
Time from last HIV test							0.123
6 months or less	76	39.8	49	35.8	27	50.0	
6–12 months	48	25.1	39	28.5	9	16.7	
More than 12 months	67	35.1	49	35.8	18	33.3	
Venue of most recent HIV test							0.417
Hospitals	129	67.5	101	68.7	38	70.4	
VCT clinics	43	22.5	34	23.1	9	16.7	
Other premises	19	9.9	12	8.2	7	13.0	
Number of HIV testing during the past 5 years							0.137^b^
1–4	177	92.7	124	90.5	53	98.1	
5–9	13	6.8	12	8.8	1	1.9	
10 or more	1	0.5	1	0.7	0	0	
Result of last HIV test							0.105
Positive	2	1.0	1	0.7	1	1.9	
Negative	178	93.2	131	95.6	47	87.0	
Not sure	11	5.8	5	3.6	6	11.1	

**Note:**

a P value from Chi-square test.

b P value from Fisher's exact test.

In Beijing, a larger proportion of participants reported having ever been tested for HIV compared with Urumqi (53.9% versus 37.2%, p = 0.001). In addition, participant preferences for HIV testing services differed significantly, with a higher proportion of participants in Beijing reporting a preference for having a fixed appointment for HIV testing as compared with participants in Urumqi (37.4% versus 22.8%, p = 0.003). There were no statistically significant differences between participants from Beijing and Urumqi in terms of HIV testing experiences.

### Motivation to seek HIV testing and response to Internet outreach

Nearly all participants (96.0%, 383/399) reported having a good or very good experience with Internet outreach, and 98.0% (391/399) reported that they would be happy to be involved in Internet outreach in the future even if reimbursement was not provided. Over three quarters of participants (79.4%, 317/399) reported being motivated to participate in the study because they were concerned about their HIV status. Nearly 40% (153/399) of men participated in the study because they were concerned about the overall health of the MSM community. Only 2.8% (11/399) of participants reported being motivated by the reimbursement. Less than 5% of participants (19/399) had heard of VCT and knew the location of at least one VCT clinic before their first sexual experience with a male. A minority (10.5%, 42/399) had ever attended a VCT clinic to receive HIV testing. Most participants (91.5%, 365/399) reported a preference for HIV testing in VCT clinics rather than hospitals. A community MSM member with health expertise was preferred (38.6%, 154/399) to represent Internet outreach services (Table 5). Most participants (80.4%, 321/399) reported that they would like the services to be available between 6–10 pm during working days, as they would have more time after work and enjoy more privacy at night.

**Table 5:** MSM's experience with Internet outreach.

Variable	Total		Beijing		Urumqi		*P* a
	n	%	n	%	n	%	
Experience with Internet outreach							0.036^b^
Very good	224	56.1	154	60.6	70	48.3	
Good	159	39.8	92	36.2	67	46.2	
Not sure	9	2.3	6	2.4	3	2.1	
Poor	5	1.3	2	0.1	3	2.1	
Very poor	2	0.5	0	0	2	1.4	
Would you use Internet outreach in the future if reimbursement not provided?							0.192 b
Yes	391	98.0	251	98.8	140	96.6	
No	4	1.0	1	0	3	4.1	
Not sure	4	1.0	2	0.1	2	1.4	
Motivation for participating in this study							0.906
Concerned about health	317	79.5	202	79.5	115	79.3	
Concerned about MSM community	153	38.4	95	37.4	58	40.0	
Opportunity to consult health professionals	83	20.8	52	20.5	31	21.4	
Financial incentive	11	2.76	8	3.1	3	2.1	
Ever heard of VCT clinics before first sex experience with a male							0.185
Yes	25	6.3	19	7.5	6	4.1	
No	374	93.7	235	92.5	139	95.9	
Aware of the location of at least one VCT clinic before first sex experience with a male							0.156
Yes	19	4.8	15	5.9	4	2.8	
No	380	95.2	239	94.1	141	97.2	
Preferred HIV testing and counseling venues							0.324
VCT clinic	365	91.5	235	92.5	130	89.8	
Hospital	34	8.5	19	7.5	15	10.2	
Preferred online Internet outreach service representative							0.003
CDC staff	84	21.1	57	22.4	27	18.6	
Clinical doctor	72	18.0	44	17.3	28	19.3	
Psychologist/psychiatrist	89	22.3	43	16.9	46	31.6	
MSM with medical background	154	38.6	110	43.3	44	30.3	

**Note:**

a P value from Chi-square test.

b P value from Fisher's exact test.

Participant preferences for Internet outreach service representative differed between Beijing and Urumqi. In Beijing, the majority of participants preferred to have an MSM with a medical background as a service provider (43.3% of Beijing participants reported this preference, versus 30.3% of Urumqi participants), while in Urumqi, more participants favored a psychologist or psychiatrist (31.6% of Urumqi participants versus 16.9% of Beijing participants).

### Passive versus active Internet outreach

More older participants responded to passive Internet recruitment, compared with younger (63.2% versus 46.2%, X^2^ = 11.400, *P* = 0.001). Those who had previously been tested for HIV were more likely to respond to passive Internet recruitment, compared with those who had never been tested for HIV (61.3% versus 51.0%, X^2^ = 4.281, *P* = 0.039). Those who had been tested for HIV more recently were more likely to respond to passive Internet recruitment, compared with those who had been tested for HIV more than 12 months prior to the study (67.7% versus 49.3%, X^2^ = 6.265, *P* = 0.012). Frequent testers (5 or more HIV tests in the past 5 years) were also more likely to respond to passive Internet recruitment, compared with those who had been tested 1–4 times in the past 5 years (67.5% versus 50.0%, X^2^ = 5.638, *P* = 0.018) (Table 6).

**Table 6:** Chi-square tests of the distribution of age and HIV testing history between participants recruited through passive routes and active routes.

	Passive recruits % (n/N)	Active recruits % (n/N)	X^2^	*P*
Age			11.400	0.001
24 years old or younger	46.2% (79/171)	53.8% (92/171)		
25 years old or older	63.2% (144/228)	36.8% (84/228)		
Ever tested for HIV?			4.281	0.039
Yes	60.9% (117/191)	39.1% (74/191)		
No	51.0% (106/208)	49.0% (102/208)		
Time from last HIV test			6.265	0.012
12 months or less	67.7% (84/124)	32.3% (40/124)		
More than 12 months	49.3% (33/67)	50.7% (34/67)		
Number of HIV tests in past 5 years			5.638	0.018
1 to 4	50.0% (34/68)	50.0% (34/68)		
5 or more	67.5% (83/123)	32.5% (40/123)		

Note: Passive recruits included participants who were recruited through posters on gay websites and word-of-mouth. Active recruits included participants who were recruited through QQ, MSN, Email, phone call or gay chat rooms.

## Discussion

More and more MSM are using the Internet to socialize and access health information [16]–[18]. Our study found that QQ, a web-based instant message service that is readily available across China, is the single most efficient online route to provide information about HIV testing and counseling services and encourage MSM to attend a testing venue. We also found that online gay chatrooms and mobile phone contact are both feasible ways to encourage MSM to seek HIV testing. While we found that e-mail is a less efficient way to encourage MSM to seek HIV testing, e-mail is a practical, low cost method of communication that merits further evaluation. Our study findings suggest that the effectiveness of different online methods of outreach may vary geographically, perhaps based on local patterns of online behavior.

Of the 3,332 contacted through active and passive outreach, 429 attended VCT clinics and 399 received HIV testing. Our response rate of 12.9% (429/3,332) is consistent with the response rates reported by previous studies that have used internet outreach to recruit individuals for health interventions. For example, Graham et al. reported that 9.1% of individuals who clicked on a website banner advertisement for smoking cessation treatment actually registered for treatment [26]. However, recruitment rates via the internet vary widely depending upon the population targeted. One recent study of a smoking cessation program among teenagers, for example, found a very low response rate of <1% [27].

The Chinese government's ‘Plan for HIV/AIDS Prevention and Control among Men Who Have Sex with Men in China, 2007–2010’ set an ambitious target of achieving a 50% or higher HIV testing rate among MSM by 2010, recommending that MSM receive HIV testing at least once per year. In our study, however, we found that the majority of MSM had not been tested for HIV in the past 12 months, and most MSM had never been tested for HIV. Rates of HIV testing were higher in Beijing than in Urumqi, with over half (53.9%) of Beijing participants and over one-third of Urumqi participants (37.2%) reporting ever having been tested for HIV. In both Beijing and Urumqi, one in three participants reported having been tested for HIV more than 12 months ago, suggesting that efforts to increase the frequency of HIV testing still need to be intensified. Most of our study participants reported that they perceive themselves to be at low or very low risk of HIV infection, though HIV prevalence in our participant population was high at nearly 5%. Increasing HIV testing efforts is essential since previous studies have shown that HIV positive MSM who are aware of their HIV status adopt safe sex behaviors in significantly higher proportions compared with MSM who are not aware of their HIV status [14], [28].

Unfortunately, while HIV VCT services are widely available across China, most MSM remain unaware of where and how to seek VCT services. Among MSM who had ever tested for HIV, more than 3 in 4 were tested in places other than VCT clinics, despite the fact that Chinese government policy mandates free HIV testing throughout the VCT system (Table 4). Unlike hospitals which have various departments and serves all types of patients, VCT clinics are especially set up for HIV testing and counseling and are supposed to provide comparatively more anonymous, specialized and confidential HIV-related services than hospitals. For these reasons, many MSM prefer to test for HIV in VCT clinics. If VCT services are publicized and tailored to the needs of MSM, these services have the potential to be a powerful platform not only for HIV testing, but also for HIV prevention efforts and linkage to care programs. One issue that we identified through our study is the lack of awareness of HIV testing services that our MSM participants reported before becoming sexually active with another male. Future efforts to reach young MSM need to include practical information on where free, anonymous HIV testing services are available. We also identified several aspects of HIV testing service delivery worth noting for future quality improvement efforts. First, we found that most MSM would like the services to be available between 6–10 pm during working days, as they would have more time after work and enjoy more privacy at night. Second, our participants reported that they would like someone from the MSM community with professional knowledge to implement Internet outreach services. Third, they reported that HIV testing services at VCT clinics would be more attractive if condoms and lubricant are available on-site. Finally, we observed geographical variations in service preferences, underscoring the importance of understanding local context in the design of HIV testing services.

In this study, two trained community members searched for contact information posted by MSM on gay websites and used this information for HIV testing outreach. The two community members each worked 4 hours per day every day for 1 month, including Saturdays and Sundays. This is a serious investment of time and energy, but one that is worthwhile in the context of high HIV prevalence among MSM. One major benefit of this active Internet outreach approach is the potential to reach younger MSM who have either never been tested for HIV or who were tested a longer time ago and/or less frequently. This is critically important since MSM who test more often tend to have less risky sexual behaviors, compared with those who test less often [29].

There were several notable strengths of this study. First, we had strong involvement from the MSM community. Our MSM volunteers found a straightforward and systematic way to reach out to MSM who had publicly posted their contact information on gay websites. Second, our study illustrates how cooperation between MSM community groups and existing government-run health services can achieve the common goal of increasing the uptake of HIV testing among MSM. Third, our study findings provide early data on how outreach and HIV testing services can be better targeted to serve the needs of the MSM community.

Several limitations are worth noting. First, our study population was recruited via the Internet, and therefore may not be representative of all MSM in the communities from which participants were recruited. Second, active Internet outreach is labor intensive, and may not be feasible across all contexts due to human resources or financial limitations. Third, we did not collect data on the number of men clicking on the online banners and forwarding study information to their peers; thus, it was impossible for us to assess the effectiveness of these two routes. Finally, due to the limitations of our study design, we were not able to compare those who responded to our internet outreach efforts and those who did not. It is important to know what types of individuals did not respond and why in order to improve the design of future internet outreach efforts, but we were not able to ascertain this in our study because we did not have the ability to identify or follow-up individuals who did not respond.

Our study findings are similar to those of previously reported research. A similar study focused on promoting HIV testing among MSM who seek male sexual partners within Internet chat rooms [22]. Researchers spent 8 hours per day over 6 months contacting MSM using Internet chat rooms. They compared the pretest and posttest data and found that self-reported HIV testing among those in the chat rooms increased from 44.5% at pretest to nearly 60% at posttest (p<0.001). Compared with our Internet outreach strategy, this intervention is more labor intensive. Other studies have documented novel approaches that aim to increase STI testing and diagnosis among MSM, such as computer alerts on electronic medical records to remind clinicians to screen for STIs during clinical consultation, and mobile phone text message reminders [30]. The US CDC has recently issued new HIV prevention guidelines that recommended the adoption of combinations of scientifically proven, cost-effective and scalable interventions targeted to the right populations in the right geographic areas, to increase the impact of HIV prevention efforts [31].

Nearly all MSM were satisfied with the Internet outreach services. They would like the services to continue and would use Internet outreach in the future, even if reimbursement is not available. Internet outreach is a promising approach for recruiting MSM, especially those who might not otherwise seek testing. Combining this strategy with other scientifically proven, cost-effective and scalable interventions that target MSM will potentially bring about even greater and longer positive impact on HIV testing among MSM. We found that the majority of MSM responding to passive recruitment have previously received HIV testing. This suggests that active recruitment approaches may be necessary to encourage very high risk MSM to get tested for HIV, and this hypothesis merits further exploration. Future studies should focus on assessing the characteristics of various online platforms, such as chat rooms, partner-seeking websites, so as to help tailor interventions to most effectively reach MSM.

## Conclusion

The MSM in China who participated in our study prefer to receive HIV testing in VCT clinics over hospital settings. Using active Internet outreach to encourage MSM to get tested for HIV at VCT clinics may be a good way to target younger, less frequently tested MSM. Scaling up Internet outreach efforts in combination with other proven strategies to increase HIV testing uptake are essential steps toward reducing HIV transmission among MSM.
